# Prediction of Dental Implants Using Machine Learning Algorithms

**DOI:** 10.1155/2022/7307675

**Published:** 2022-06-20

**Authors:** Mafawez T. Alharbi, Mutiq M. Almutiq

**Affiliations:** ^1^Department of Natural and Applied Sciences, Applied College, Qassim University, Buraydah, Saudi Arabia; ^2^Department of Management Information Systems and Production Management, College of Business and Economics, Qassim University, Buraydah, Saudi Arabia

## Abstract

It has been claimed that artificial intelligence (AI) has transformative potential for the healthcare sector by enabling increased productivity and creative methods of delivering healthcare services. Recently, there has been a major shift to artificial intelligence by businesses, government, and private sectors in general and the health sector in particular. Many studies have proven that artificial intelligence is contributing greatly to the health sector by discovering diseases and determining the best treatments for patients. Dentistry requires new innovative methods that serve both the patient and the service provider in obtaining the best and appropriate medical services. Artificial intelligence has the ability to develop the field of dentistry through early diagnosis and prediction of dental implant cases. This research develops a set of four machine learning algorithms to predict when a patient might need dental implants. These models are the Bayesian network, random forest, AdaBoost algorithm, and improved AdaBoost algorithm. This work shows that the developed algorithms can predict when a patient needs dental implants. Also, we believe that this proposal will advise managers and decision-makers in targeting patients with particular diagnoses. Analysis of the obtained results indicates good performance of the developed machine learning. As a result of this research, we note that the proposed improved AdaBoost algorithm increases the level of prediction accuracy and gives significantly higher performance than the other studied methods with the accuracy for the improved AdaBoost algorithm reaching 91.7%.

## 1. Introduction

Artificial intelligence (AI), as one of the newest fields of computer science, has been extensively and formally researched since the 1950s. John McCarthy, one of the founding fathers of AI, defined it as “the science and engineering of making intelligent machines” [1]. Significant transformations in the public and private sectors at the level of reinnovation in business models use artificial intelligence techniques with customer experience contributing to more effective decisions [2]. Applications of AI can be found in a variety of fields. The past several years have seen a significant increase in the use of artificial intelligence in healthcare with promising outcomes. Human biology and dental implants are just a few of the healthcare fields in which artificial intelligence (AI) has already found application [3–5].

Interpretation of medical data for automated analysis is the subject of two case studies [6]. In the first case study, based on cognitive test results and demographic data, Bayesian inference, a machine learning technique, was used to diagnose Alzheimer's disease. Artificial neural networks (ANNs) were used in the second case study for the automatic classification of breast cancer cell pictures [6]. Many studies have confirmed that the use of artificial intelligence allows for the ability to improve the diagnoses and treatment of patients and thus take full advantage of this technology within the medical environment [7–10]. Dental clinics have presented several models and techniques designed to provide medical consultations and determine the patient's dental condition [7].

It is essential to use technology that contributes to improving quality while maintaining costs in a dental clinic. Otherwise, misdiagnosis may result in expensive litigation, thereby increasing the expenses of the dental clinic [9]. A new approach for diagnosing the treatment of dental caries using the Bayesian machine learning algorithm was proposed [11]. A Bayesian network is designed to provide decision support among different treatment plans. Using this method, the dentist can treat patients with an increased level of confidence and an overall improvement in performance. The Bayesian network provides a strong mathematical foundation for tackling such problems.

This research contributes to identifying patients who may need dental implants in a timely manner. As government hospitals and private health clinics are overcrowded, there may be a very long waiting list for patients to obtain dental implants. Therefore, there is a need to prepare a scientific research proposal using an artificial intelligence technique.

The main contributions of the current work are to use four machine learning algorithms, namely, the Bayesian network, random forest, AdaBoost algorithm, and improved AdaBoost algorithm to predict patients who are expected to need dental implants by relying on previous data and current symptoms. The accuracy of all algorithms is presented and shown in a graph.

### 1.1. Related Work

In the field of healthcare, scientists have published a few scientific studies that use artificial intelligence based on machine learning algorithms and successfully linked them to real life [8, 12, 13]. Over the past few years, scientific publication in the field of medical artificial intelligence has increased nearly tenfold, as individual predictions of short-term diseases provide appropriate outcomes for multiple conditions including diabetes, cancer, heart, and mental illness [4, 14].

Reducing dependence on human decision-making and automation of repetitive tasks, as one of the most important uses of artificial intelligence, has been accomplished in many sectors. According to a recent study [2], the healthcare sector accounts for a substantial portion of public spending, and the use of artificial intelligence applications in healthcare and medical research has expanded significantly.

Bayesian networks are proposed [15] as a decision-support tool in public healthcare systems. This article introduces LARIISA Bay, a novel component based on Bayesian networks that works in conjunction with LARIISA. It is a sophisticated platform that enables the development of applications in the field of public health systems. The suggested system's primary purpose is to assist health teams in diagnosing diseases more accurately by utilizing data obtained from LARIISA users.

Machine learning models of data complexity and diversity in health sector applications have directly and indirectly contributed to the ability to predict diseases early. Heart disease, for example, is one of the most lethal diseases. A large number of researchers around the world are using data from heart disease patients to anticipate or predict this disease and, as a result, prevent the untimely death of many people. Machine learning algorithms are an effective tool for classification and prediction tasks [8, 12].

Reliance on information systems in most dental clinics is increasing. The focus is on providing logistical and administrative support to facilitate and automate administrative functions such as appointment alerts and bills [9]. Clinicians' diagnostic practices have improved as a result of these modifications. For this reason, there is a need to uncover new technologies that can assist in the development of an undeveloped medical area such as clinical decision support [16]. This technology has the ability to enhance patient care by going beyond administrative tasks and providing personalized advice based on the patient's specific medical and dental needs [9, 17].

In the coming decades, due to the acceleration of technological progress, much manual work will be automated [7, 16]. Dentistry is expected to witness a remarkable shift in the automation of simple routine tasks and the support of dental medical staff; this shift will contribute to improving quality [8]. We concur that technology will not replace dentists but will rather complement and support dentists in providing the greatest possible patient experiences and treatments.

Dental implants have a very high success rate for replacing lost teeth. Dental implants are in high demand, and this need is growing rapidly [18].

According to Revilla-León [19], artificial intelligence techniques have contributed to the development of osteosynthesis prediction models to predict implant success and therefore improve implant designs. Artificial intelligence is speedily affecting healthcare, and this technology will perform key roles in strategically and intelligently supporting diverse medical functions [20].

Machine learning algorithms for predicting the success of dental implants have been studied in [18]. The following algorithms were put to the test: neural networks, support vector machines, k-nearest neighbors, and a newly developed technique known as nearest neighbors with structural risk minimization (NNSRM).

A Bayesian network was used to develop a clinical decision support system for the treatment of modern dental caries [21]. Using the most recent results and conclusions in pathology, the initial version of the plan was drafted. The proposed result is compatible with search predictions based on well-defined situations. In the coming stages, the four machine learning algorithms studied will be validated using data.

The random forest classifier was shown to be the most effective method for achieving the greatest outcomes [22]. With this approach, it is possible to see how a number of different feature selection strategies can be used to increase classification accuracy and to ensure that the features selected are those most relevant to the problem at hand. Dental implant data were searched for thresholds using a random forest classifier. The chosen threshold value was found to be optimal for classification accuracy, as it outperformed all other classifiers [22]. AdaBoost and bagging are compared [23]. The results demonstrate that classifier ensembles can increase prediction performance, although the bagging technique outperforms the AdaBoost technique [24]. Liu et al. [23] examined the prediction rate of dental implant treatment using numerous supervised learning methodologies including AdaBoost techniques to classify clinical data. It was observed that using supervised learning techniques successfully evaluated the failure percentage of dental implant treatment using the data [23].

## 2. Methodology

The methodology in this research consists of two stages. The first stage is conducting the survey, and the second stage is applying machine learning algorithms.

### 2.1. Survey

Surveys are probably the most commonly used research method for many sectors [25]. Based on the opinion of dental specialists, there are behavioral factors for patients that directly affect the implant of teeth. As health data are highly sensitive, surveys are a good option for obtaining data in this sector. In addition, surveys are widely used in software engineering.

In this research, six significant factors that affect the dental composition of patients have been identified. These factors were identified through previous studies, as well as by conducting several interviews with dental specialists. As data for these factors are not available in the databases in many clinics, surveys were used in this research to collect these data.

### 2.2. Machine Learning Algorithms

Artificial intelligence is an umbrella term for many topics. Machine learning (ML) algorithms are considered a subtopic of AI. Some ML algorithms are *K*-means, SVM, logistic regression, random forest, Bayesian network, and AdaBoost. This research will use the following ML algorithms: Bayesian network, random forest, and AdaBoost. In addition, the research has developed a new algorithm of AdaBoost called “improved AdaBoost algorithm.” We present below a short description of each machine learning algorithm used in this study.

The BN is a highly useful model for depicting and modeling current knowledge to better understand and perceive uncertainties and complexities [26]. The following stages must be completed in order to build an effective BN model: identify the factor, draw the BN model, parametrize the model, and apply the inference algorithm. The correctness of any inference in BN is guaranteed, and the model incorporates prior knowledge with the observed data. The technique allows situations to be handled even when some data are missing. There is flexible modeling of features via hierarchical models when correct and reliable statistical data have been collected. This technique has the ability to deal with random variables or inaccurate knowledge. Bayes' theorem, which was devised by Reverend Thomas Bayes in the eighteenth century, allows us to deduce the likelihood of a cause from the observation of its effect. Bayesian networks [27] are graphical structures that are used to represent the interactions between these two variables. Bayesian networks are able to present the uncertainties from current and previous data. These networks are used to factorize a joint probability by spreading a group of random variables [28]. They are described as graphical representations of random variables connected by arrows that signify a dependency.

Bayesian networks are divided into two branches of traditional Bayesian networks, namely, static Bayesian networks and dynamic Bayesian networks. Due to the statistical properties contained in the training data, the Bayesian technique may perform more accurately than the classic point estimation method in complex regression and classification problems [29]. The Bayesian approach is useful since it guarantees the validity of all conclusions, and the BN model incorporates prior information into the observed data. The technique enables situations to be handled in the absence of some data. When accurate and reliable statistical data are acquired, it is possible to model features in a flexible manner using hierarchical models. This technique is capable of dealing with unpredictable factors and insufficient knowledge. BNs can be used to describe how a solution is arrived at [30].

The random forest algorithm works on the principle of ensembles. This algorithm combines a group of weak learners in a parallel way [31]. Each individual learner is trained by a random subset of the data. Then, the outputs of all learners are averaged to build a strong prediction rule. For weak learners, decision trees with a depth of one are most commonly used. These decision trees are also known as decision stumps. Random forest, which has been widely used in classification and prediction, and has several advantages compared with other machine learning algorithms. Therefore, random forest is used in a large scope of applications [32].

In contrast with the random forest algorithm, the AdaBoost algorithm uses multiple base learners in a sequential process to predict the results [33]. Each individual learner attempts to correct the errors of its predecessor. First, a learner is built from training data in which observations are given equal weights. The weight value indicates how each observation is significant regarding the classification [34]. Afterwards, the next learner is built which tries to correct the errors present in the first learner. Thus, at every iteration, more weight is given to the observations that are predicted incorrectly. Hence, the weights of the misclassified data points are increased and the weights of the ones predicted correctly are lowered. The training weight values are normalized after all misclassified observations are updated. This process is iterated and learners are added until the complete training dataset is predicted correctly or the maximum number of learners is reached [35].

### 2.3. Proposed System

The aim of this research is to study some interesting machine learning algorithms for the prediction of dental implants. The focus of this research is on ensemble learning algorithms. The following four most popular algorithms are considered: Bayesian network, random forest, AdaBoost, and improved AdaBoost. The results given by the studied algorithms are compared and discussed. In addition, this study proposes a new improvement of the standard AdaBoost classifier to increase its prediction capability. This modification optimizes the sample weights parameter to initialize the AdaBoost algorithm. Note that in the literature, AdaBoost typically uses a discrete uniform distribution for the initialization weights. The sample weights are a set of weights that specifies the value of each sample. It is known that AdaBoost is extremely sensitive to noisy data and outliers. Hence, by using an optimal initialization for the sample weights parameter, the research expects to find improvement in prediction ability.

### 2.4. First Algorithm: Bayesian Network

A Bayesian network is a probabilistic graphical model that measures the conditional dependence structure of a set of random variables based on the Bayes theorem. This model consists of two major parts: a directed acyclic graph and a set of conditional probability distributions. Let *Y* denote the response variable which has *k* possible outcomes. *X* are the features that characterize *Y*. Using the Bayes theorem, the conditional probability of each outcome, given *X*, is of the following form:

(1) $$\begin{array}{c} P\left(Y/X\right)=\frac{P\left(X/Y\right)P\left(Y\right)}{P\left(X\right)}, \end{array}$$

where *P(Y)* is the prior distribution of parameter *Y*; *P(Y/X)* is the posterior distribution, the probability of *Y* given new data *X*; and *P(X|Y)* is the likelihood function, the probability of *X* given existing data *Y*.

To make predictions using the Bayesian network, there are four stages: identify the factor, draw the BN model, parametrize the model, and finally apply inference algorithms. These stages are discussed.

#### 2.4.1. Stage One: Identify the Factor

In this section, we identify some major factors which have a direct effect on when the patient will require dental implants. The following six factors were identified by interviews and the literature review: age of patient, level of care for the teeth, Dental crowns, type of food, patient's healthcare insurance, and patient's other diseases.  Table 1 provides the factors with their states.

#### 2.4.2. Stage Two: Draw the BN model

This section presents the relationship between the selected factors in stage 1. These factors have been fused together to draw the BN model. The following BN tools are used to build the BN model, namely, Bayes Net Toolbox, MATLAB, and GeNIe. This research has chosen GeNIe tools because they are fast and free to download; in addition, GeNIe supports graphical user interface. GeNIe is a development environment that has the ability to build graphical decision theoretic models. University of Pittsburgh's Decision Systems Laboratory has been developing this tool since 1995 [36].

Six variables were identified, and then the causal relationships between these variables (nodes) were defined. In order to draw the proposed model, an abbreviation is suggested for each factor.  Table 2 provides the abbreviations for the chosen factors.

The BN model is presented using GeNIe tools as shown in Figure 1. The model consists of six nodes. The main node, called “PredictionDI,” is used to predict, whereas the other nodes affect the main node and are called Age, DentalC, CareL TypeF, Insurance, and Diseases.

Expert knowledge and historical data can be incorporated in the suggested model to obtain the network's joint probability distribution.

#### 2.4.3. Stage Three: To Parametrize the Model

To parametrize the BN model, a survey was created. This survey consists of seven questions, as shown in Figure 1. The survey was created by Google survey and distributed in the Qassim region of Saudi Arabia.

(1) What is your age?
  - Under 20
  - Between 20 and 40
  - Over 40
(2) Have you had dental implants in the past?
  - Yes
  - No
(3) Have you had dental crowns in the past?
  - Yes
  - No
(4) What is the level of care for your teeth?
  - Always
  - Sometimes
  - Rarely
(5) What is your food type?
  - Heathy
  - Nonhealthy
(6) Do you have health insurance?
  - Yes
  - No
(7) Do you have any other disease?
  - Yes 
  - No

The correctness of the learned network depends on the amount of training data available to improve the accuracy of the learned model. One hundred and seven participants participated in the survey. The Excel file contains the result of the survey. To import the Excel file to the chosen tool (GeNIe), the Excel file needed to be converted to text file and saved in Notepad.

Figure 2 shows the data file opened by the GeNIe tool. Now, we have reached the stage of matching the result of the survey (data file) with the proposed BN model. The tool has the automatic ability to identify the name of each column and match it with the data file, as shown in Figure 3. It is evident that one column, “Timestamp,” is not matched.

The final step in this stage is to apply parameter learning action to learn from the data, as shown in Figure 4. This proves that the parameter learning has been completed.

For example, the state of the node named “CarL” is shown in Figure 5. This shows the probability of each state in CareL node. Expert projections for all probable and current diagnoses are translated into conditional probabilities in this probability table.

#### 2.4.4. Apply Inference Algorithm

Inference in this network entails determining the selected variable's conditional probability given that other variables are instantiated to particular values. For example, when we need to compute the probability of predicting the dental implant, given some diagnoses for the patients, cases 1, 2, and 3 present these situations.

The polytree algorithm has been chosen for this model as one path between two nodes. This section presents three cases of using the proposed BN model, with each case having a different state of factors.

In case 1, an evidence node has been observed. Observed nodes become instantiated, which indicates that their outcome is known with certainty in the basic case. Evidence for each factor must be identified in order to predict the dental implant. The evidence entered is marked by underlining the state and showing the bar to be 100% (Figure 6).  Table 3 provides the chosen evidence for each node.

Based on the evidence given in Table 1 and the previous data (survey), the BN model in Figure 7 shows the prediction of dental implant for the patient. The patient's probability of requiring dental implant is 0.9 because all the states of each factor affecting the dental implant are very high. The probability of the patient not requiring dental implant is 0.1.

Case 2 presents different states for each factor. The evidence here differs from the first case.  Table 4 provides the states for each factor.

This evidence is applied to the BN model and the inference is applied. The result for the inference is shown in Figure 8. The patient probability of requiring dental implant is 0.166; this means that with the entered evidence, the prediction for the patient requiring dental implant is very low. However, the probability of the patient not requiring dental implant is 0.833. As a result, the prediction for the patient to not require dental implant is very high.

In case 3, BN can also deal with missing values. For example, we assume that two of the six factors are missing, namely, DentalC and other diseases, whereas the rest of the factors are known, namely, age, care level, food type, and healthcare insurance. This is given in Table 5.

In Figure 9, it is clear that the two factors with missing values have a question mark (?) underneath the node, namely, DentalC and Diseases. 

These factors with missing values are applied to the BN model, and the result for the inference is shown in Figure 10. The probability of the patient requiring dental implant is 0.213, which means that based on the entered evidence, the likelihood for the patient requiring dental implant is very low. However, the patient probability to not require dental implant is 0.786. As a result, the prediction for the patient to not require dental implant is very high.

We consider now the overall dataset and obtain an accuracy of 72.8%.  Figure 11 shows the screenshot for the prediction accuracy result given by the BN algorithm.

### 2.5. Second Algorithm: Random Forest

This model is built from a training set {(*x*_*i*_, *y*_*i*_)}_*i*=1_^*N*^ that predicts *Y* for a new observation *X* formalized by a weight function *W*:

(2) $$\begin{array}{c} Y=\sum_{i=1}^{N}W\left(x_{i},X\right)\;y_{i}, \end{array}$$

where *W*(*x*_*i*_, *X*) is the nonnegative weight of the *i*^*th*^ training observation relative to the new observation *X* in the same learner.

As random forest averages the predictions of a set of all *M* learners with individual weight functions *W*_*j*_, its prediction is given by

(3) $$\begin{array}{c} Y=\sum_{i=1}^{N}\left(\frac{1}{M}\overset{M}{\underset{j=1}{\sum }}w_{j}\left(x_{i},X\right)\right)y_{i}. \end{array}$$

Random forest has been applied to dental implants prediction. The authors implement and test this algorithm on the dental implant dataset. The dataset is randomly split into training and testing sets to assign two-thirds of the data points to the former and the remaining one-third of the data points to the latter. The efficiency of the model's prediction is evaluated by the accuracy, which is the percentage of correct predictions. Accuracy is found to be above 77.8%. This moderate prediction capability is acceptable, since the random forest model is very sensitive to outliers and nonlinear data.

Figure 12 shows the screenshot for the prediction result given by the random forest algorithm applied on the test dataset in Python program language.

Two cases of using random forest are presented and each case has a different state of factors. In case 1, the random forest algorithm has been applied to the prediction of the dental implant dataset. The chosen evidence for case 1 here is the same as what has been described previously in Table 3. Based on the training dataset, the RF model indicates that the prediction of dental implant for case 1 takes the value “No.” This means that the patient in this case does not require dental implant, and all the states of each factor do not indicate dental implant. The chosen evidence for case 2 is the same as that which has been described previously in Table 4. Case 2 presents different states for each factor. The prediction value calculated by the RF model is also equal to “No.”

### 2.6. Third Algorithm: AdaBoost Algorithm

A boosted classifier is a classifier of the form

(4) $$\begin{array}{c} Y_{M}\left(X\right)=\sum_{m=1}^{M}f_{m}\left(X\right), \end{array}$$

where each *f*_*m*_(*X*) is a weak learner that takes an observation *X* as input and returns a value indicating the class of the observation. Each weak learner produces an output hypothesis *h()* which fixes a prediction *h*(*x*_*i*_) for each sample in the training set. At each iteration *m*, a weak learner is selected and assigned a coefficient *α*_*m*_ such that the total training error *E*_*m*_ of the resulting boosted classifier is minimized.

(5) $$\begin{array}{c} E_{m}=\sum_{i}E\left[Y_{m-1}\left(x_{i}\right)+\alpha_{m}h\left(x_{i}\right)\right]. \end{array}$$

The AdaBoost algorithm has been applied to the prediction of dental implants. We implement and test this algorithm on the dental implement dataset. We implement and test this algorithm on the dental health care dataset. We receive an accuracy of 86.1 percent, which is higher than the accuracy of random forest.

Figure 13 shows a screenshot of the prediction result obtained by the standard AdaBoost algorithm applied to the dental health care dataset in Python program language.

Similar to the RF model, two cases of using the AdaBoost algorithm are presented with the result. Each case has a different state of factors.

In case 1, the research tests the AdaBoost algorithm with the specific case given in Table 3. Based on the same training dataset, the AdaBoost algorithm indicates that the prediction of dental implant for case 1 is “No.” This means that the patient in this case does not need dental implant.

In case 2, the research tests the AdaBoost algorithm with the specific case given in Table 4. The prediction value given in this case is also equal to “No.” Note that these results coincide with those given by the RF model but not with the BN predictions. This could be explained by the use of nonoptimal sample weights initialization.

### 2.7. Fourth Algorithm: Improved AdaBoost Algorithm

As the AdaBoost algorithm tries to correct misclassified data points in the training set, one has to be careful with outliers or noise. Indeed, these outliers or wrong examples will distort the prediction and lead to a poor algorithm performance. For this reason, each data point has a different impact on the prediction accuracy. Therefore, to lead better performance, we also propose to modify the traditional AdaBoost algorithm. The improved AdaBoost algorithm is initialized by a random sample weight. Hence, instead of assigning an equal weight to each data point for the sample set initialization, we suggest running the AdaBoost algorithm with different random sample weight values and keeping the initialization that gives the higher level of accuracy. By using more suitable sample weights, we expect to obtain better prediction accuracy. In the following section, we describe the pseudocode of the modified AdaBoost version.

## 3. Implementations and Results

Let us test our implementation for the improved AdaBoost algorithm on the dental healthcare dataset and compare its predictive power with the other studied classifiers. We use the dental healthcare dataset as we have done with the previously presented machine learning algorithms. This dataset is shown in Figure 14.

The accuracy of the classifier is used as a performance measurement to express the prediction ability of the algorithm. The accuracy will tell us how many times the algorithm predicts the correct classes. Improved AdaBoost reached an accuracy of 91.7%, which is higher than the accuracy of the standard AdaBoost method. The predictive power of the improved model is really significant.

Figure 15 shows a screenshot of the prediction result given by the improved AdaBoost algorithm applied to the dental healthcare dataset.

We applied the improved AdaBoost model to the two specific cases just as we did with the previous prediction models. The result for the inference is summarized by the following two cases. The prediction of case 1 is equal to “Yes.” Hence, the patient might need dental implant. However, the patient in case 2 does not require dental implant since the prediction result is “No.” Note that these results coincide with those given by the BN model. These results confirm the effectiveness of the improved Table 6 AdaBoost algorithm.

Table 6 provides the comparison results between the proposed methods and the other studied machine learning algorithms on the overall dataset. Note that the proposed method gives a higher level of accuracy.  Figure 16 shows the effectiveness of the proposed method.

From this experimental study, we note that the proposed improved AdaBoost algorithm increases the prediction accuracy and gives significantly higher performance than the other studied methods. This successful capability can provide a powerful tool for enhancing the prediction of dental implant. This gain in performance is due to the optimal weights initialization procedure we propose in this work.

## 4. Discussion

Recent years have seen an upsurge in the use of artificial intelligence in implant dentistry. The article [19] conducts a comprehensive evaluation to assess the application of artificial intelligence to implant dentistry in terms of implant type recognition, implant success strength, and optimal implant design. The review of this approach makes use of two databases, including PubMed and Scopus. One study that used k-nearest neighbors (*k*-NN) found that the most frequently used AI models were regression analysis (support vector machine classification), decision tree learning, logistic regression, and classifier neural network.

In addition, Mclachlan et al. [37] presented a demonstration of CardiPro which is an online application characterized by flexibility and interaction with BN models. This application was designed to facilitate the use of Bayesian technology for nontechnical users such as patients and doctors. CardiPro calculates probabilities in real time. CardiPro, which was developed as an offshoot of the PamBayesian Research Project (https://www.pambayesian.org), is considered one of the first applications to depend on Bayesian technology. It is used to support medical decisions based on artificial intelligence.

Nevertheless, to the best of our knowledge, there is no research paper in the literature that uses the four machine learning algorithms which are presented in this research to predict dental implant. As a result, this research contributes to the identification of patients who may require dental implants in a timely manner, as the government hospitals and private health clinics are overcrowded and there may be a very long waiting list for patients to obtain dental implants.

This research presented a highly useful model for depicting and modeling current knowledge to better understand and perceive uncertainties and complexities. As a result, this will help equip managers and decision-makers to target patients who have these diagnoses. In addition, the results of the research are useful in preparing and processing the materials needed for dental implants and knowing the future health needs in the public and private sector.

From empirical evaluation of the BN, random forest, AdaBoost algorithm, and improved AdaBoost algorithm, four different algorithms are trained and tested on a dental implement dataset to obtain their respective prediction accuracy.

In BN, the correctness of any inferences is guaranteed and incorporates prior knowledge to the observed data. BN allows situations to be handled even when some data are missing with flexible modeling of features via hierarchical models when correct and reliable statistical data have been collected. This technique has the ability to deal with random variables or inaccurate knowledge.

Obtained results revealed that the improved AdaBoost algorithm outperforms the baseline AdaBoost algorithm and the random forest algorithm in terms of accuracy. As we used a more suitable sample weight value that relies on the studied real-life dataset, the prediction accuracy of the improved AdaBoost algorithm is significantly enhanced. Therefore, it is important to search for the optimal sample weight initialization to increase the predictive power of the AdaBoost algorithm.

In addition, when applying the random forest classifier, we obtain a moderate level of accuracy in comparison with the improved AdaBoost algorithm that achieves better performance. This result may be explained by the fact that the random forest algorithm considers the average or the majority of the predictions made by each base learner. However, when using the AdaBoost algorithm, every base learner contributes a varying amount to the final prediction.

Moreover, adapting a new technology to a new environment is difficult, and medical applications are extremely costly [16]. There are significant challenges and limitations in this research, the most important of which is data acquisition and access to the database of healthcare in general and dental patients in particular. This limitation might be due to the privacy and security of patient data. Some clinics do not have sufficient information about their patients, and the data in most cases are incomplete and not well-structured. In addition, we consider preserving the privacy of sensitive data as discussed in [38] as part of our future enhancements.

## 5. Conclusions

This research presents four machine learning algorithms to predict the requirement of dental implants by gathering patient diagnoses and importing the data to machine learning technology. As a result, the proposed model in this research has the ability to predict when patients might require dental implants through the use of machine learning technology which depends on patients' historical data and current symptoms. We believe that this proposal will advise dentists and decision-makers in targeting patients with particular diagnoses.

The empirical comparison presented shows that the improved version of the AdaBoost algorithm gives higher accuracy. Such improvement in correct decision-making may reduce risks of dental implant problems. Our proposal is based on the optimization of the sample weights initialization parameter. This finding contributes to the research community. Indeed, we recommend the employment of a more efficient iterative process for the sample weights AdaBoost initialization instead of setting its value ad hoc to the uniform distribution. In conclusion, the AdaBoost algorithm appears to be very sensitive to noise. Hence, the prediction efficiency of this algorithm is clearly influenced by considering the optimal initialization sample weights that should be related to a specified dataset.

In future work, we need to study the determination of the optimal sample weights along with the optimization of the other hyperparameter AdaBoost algorithm such as the number of base learners, the learning rate, the random state, and the maximum depth of the individual learner. In addition, our future work will add more diagnoses and collect more data to feed the AI algorithms. Also, different machine learning algorithms will be used. We also intend to test the proposed method on other type of datasets and study its computational complexity.

## Figures and Tables

**Figure 1:** BN model.

**Figure 2:** Data file.

**Figure 3:** Column matching.

**Figure 4:** Parameter learning.

**Figure 5:** Conditional probabilities table.

**Figure 6:** Setting the evidence.

**Figure 7:** BN prediction for case 1.

**Figure 8:** BN prediction for case 2.

**Figure 9:** Missing values.

**Figure 10:** BN prediction for case 3.

**Figure 11:** BN accuracy of all cases.

**Figure 12:** Prediction accuracy of the random forest algorithm.

**Figure 13:** Prediction accuracy of the standard AdaBoost algorithm.

**Figure 14:** A random sample of examples from the dental healthcare dataset.

**Figure 15:** Prediction accuracy of the improved AdaBoost algorithm.

**Figure 16:** Graph of prediction accuracy values achieved by different machine learning methods.

**Algorithm 1:** Improved AdaBoost pseudocode.

**Table 1:** Factors with their states.

No.	Factor	State 1	State 2	State 3
1	Age	Under 20	Between 20 and 40	Over 40
2	Dental crowns	Yes	No	
3	Care level	Always	Sometimes	Rarely
4	Type of food	Healthy	Non_healthy	—
5	Healthcare insurance	Yes	No	—
6	Other diseases	Yes	No	—

**Table 2:** Factor abbreviations.

No.	Factor	Factor abbreviation
1	Age	Age
2	Dental crowns	DentalC
3	Care level	CareL
4	Type of food	TypeF
5	Healthcare insurance	Insurance
6	Other diseases	Diseases
7	Prediction dental implant	PredictionDI

**Table 3:** Chosen evidence for case 1.

No.	Factor	State 1
1	Age	Over 40
2	DentalC	Yes
3	Care level	Rarely
4	Type of food	Nonhealthy
5	Healthcare insurance	Yes
6	Other diseases	No

**Table 4:** Chosen evidence for case 2.

No.	Factor	State
1	Age	Under 20
2	DentalC	No
3	Care level	Always
4	Food type	Healthy
5	Healthcare insurance	No
6	Diseases	No

**Table 5:** Chosen evidence for case 3.

No.	Factor	State
1	Age	Under 20
2	DentalC	—
3	Care level	Always
4	Food type	Healthy
5	Healthcare insurance	No
6	Diseases	—

**Table 6:** Accuracy comparison result.

Methods	Bayesian network (%)	Random forest (%)	AdaBoost (%)	Proposed method (improved AdaBoost) (%)
Accuracy	72.8	77.8	86.1	91.7

## Data Availability

The data used to support this study are available from the corresponding author upon request.

## References

[1] Reddy S., Fox J., Purohit M. P. (2019). Artificial intelligence-enabled healthcare delivery. *Journal of the Royal Society of Medicine*.

[2] Alshahrani A., Dennehy D., Mäntymäki M. (2021). *An Attention-Based View of AI Assimilation in Public Sector Organizations: The Case of Saudi Arabia*.

[3] Takahashi T., Nozaki K., Gonda T., Mameno T., Wada M., Ikebe K. (2020). Identification of dental implants using deep learning-pilot study. *International Journal of Implant Dentistry*.

[4] Beede E., Baylor E., Hersch F. A human-centered evaluation of a deep learning system deployed in clinics for the detection of diabetic retinopathy.

[5] Akhtar S. M., Nazir M., Saleem K. (2022). A multi-agent formalism based on contextual defeasible logic for healthcare systems. *Frontiers in Public Health*.

[6] Maity N. G., Das S. Machine learning for improved diagnosis and prognosis in healthcare.

[7] Sunarti S., Fadzlul Rahman F., Naufal M., Risky M., Febriyanto K., Masnina R. (2021). Artificial intelligence in healthcare: opportunities and risk for future. *Gaceta Sanitaria*.

[8] Pallathadka H., Mustafa M., Sanchez D. T., Sekhar Sajja G., Gour S., Naved M. (2021). Impact of machine learning on management, healthcare and agriculture. *Materials Today Proceedings*.

[9] Goh W. P., Tao X., Zhang J., Yong J. (2016). Decision support systems for adoption in dental clinics: a survey. *Knowledge-Based Systems*.

[10] Javed S., Zakirulla M., Baig R. U., Asif S. M., Meer A. B. (2020). Development of artificial neural network model for prediction of post-streptococcus mutans in dental caries. *Computer Methods and Programs in Biomedicine*.

[11] Bhatia A., Singh R. (2013). Using Bayesian Network as Decision making system tool for deciding Treatment plan for Dental caries. *Journal of Academia and Industrial Research (JAIR)*.

[12] Ahmed R., Nasiri F., Zayed T. (2021). A novel Neutrosophic-based machine learning approach for maintenance prioritization in healthcare facilities. *Journal of Building Engineering*.

[13] Barmak B. A., Galluci G. O., Att W., Dent M. Artificial Intelligence Applications in Implant Dentistry. *A Systematic Review*.

[14] Osman Andersen T., Nunes F., Wilcox L., Kaziunas E., Matthiesen S., Magrabi F. Realizing AI in healthcare: challenges appearing in the wild.

[15] Teles G., Oliveira C., Braga R. Using Bayesian networks to improve the decision-making process in public health systems.

[16] Grischke J., Johannsmeier L., Eich L., Griga L., Haddadin S. (2020). Dentronics: towards robotics and artificial intelligence in dentistry. *Dental Materials*.

[17] Nasseef O. A., Baabdullah A. M., Alalwan A. A., Lal B., Dwivedi Y. K. (2021). *Artificial Intelligence-Based Public Healthcare Systems: G2G Knowledge-Based Exchange to Enhance the Decision-Making Process*.

[18] Oliveira A. L. I., Baldisserotto C., Baldisserotto J. A comparative study on machine learning techniques for prediction of success of dental implants.

[19] Revilla-León M., Gómez-Polo M., Vyas S. (2021). Artificial intelligence models for tooth-supported fixed and removable prosthodontics: a systematic review. *The Journal of Prosthetic Dentistry*.

[20] LaRosa E., Danks D. Impacts on trust of healthcare AI.

[21] Bessani M., Lins E. C., Delbem A., Maciel C. Construction of a clinical decision support system for dental caries management using BN.

[22] Ganz N., Ares A. E., Kuna H. D. (2021). Procedure to improve the accuracy of dental implant failures by data science techniques. *Journal of Computer Science and Technology*.

[23] Liu C.-H., Lin C.-J., Hu Y.-H., You Z.-H. (2018). Predicting the failure of dental implants using supervised learning techniques. *Applied Sciences*.

[24] Alarifi A., AlZubi A. A. (2018). Memetic search optimization along with genetic scale recurrent neural network for predictive rate of implant treatment. *Journal of Medical Systems*.

[25] Mathers, Joseph N., Fox N. J., Hunn A. (1998). *Surveys and questionnaires*.

[26] Carriger J. F., Yee S. H., Fisher W. S. (2019). An introduction to Bayesian networks as assessment and decision support tools for managing coral reef ecosystem services. *Ocean & Coastal Management*.

[27] Richard E. (2009). Neapolitan,Chapter 5 - foundations of bayesian networks. *Richard E. Neapolitan,Probabilistic Methods for Bioinformatics*.

[28] Koller D., Friedman N. (2009). *Probabilistic Graphical Models: Principles and Techniques*.

[29] Morales J., Yu W. (2021). Improving neural network’s performance using Bayesian inference. *Neurocomputing*.

[30] Alharbi M., Platt A., Al-Bayatti A. H. (2013). Personal Learning Environment.

[31] Sarica A., Cerasa A., Quattrone A. (2017). Random forest algorithm for the classification of neuroimaging data in alzheimer’s disease: a systematic review. *Frontiers in Aging Neuroscience*.

[32] Liu Y., Wang Y., Zhang J. New machine learning algorithm: random forest Information Computing and Applications.

[33] Cao Y., Miao Q. G., Liu J. C., Gao L. (2014). Advance and prospects of AdaBoost algorithm. *Acta Automatica Sinica*.

[34] Schapire R. E. (2013). Explaining adaboost. *Empirical Inference*.

[35] Chengsheng T., Huacheng L., Bing X. AdaBoost typical Algorithm and its application researchMATEC Web of Conferences.

[36] BayesFusion D. A. (2021). Modeling, Decision Support. https://www.bayesfusion.com/genie/.

[37] Mclachlan S., Paterson H., Dube K. Real-time online probabilistic medical computation using bayesian networks.

[38] Arikumar K. S., Prathiba S. B., Alazab M. (2022). Fl-pmi: federated learning-based person movement identification through wearable devices in smart healthcare systems. *Sensors*.

